This article has been retracted.

# Effects of microRNA-211 on proliferation and apoptosis of lens epithelial cells by targeting *SIRT1* gene in diabetic cataract mice

**DOI:** 10.1042/BSR20170695

**Published:** 2017-07-27

**Authors:** Kun Zeng, Qi-Gao Feng, Bao-Tao Lin, Da-Hui Ma, Chun-Min Liu

**Affiliations:** Shenzhen Key Laboratory of Ophthalmology, Shenzhen Eye Hospital, Ophthalmology College of Shenzhen University, Shenzhen 518000, P.R. China

**Keywords:** Apoptosis, Diabetic cataract, Lens epithelial cells, microRNA-211, Proliferation, SIRTI

## Abstract

Our study aimed at exploring the effects of *miR-211* on the proliferation and apoptosis of lens epithelial cells in diabetic cataract mice by targetting NAD^+^-dependent histone deacetylase sirtulin 1 (SIRT1). Healthy male mice were assigned into normal and diabetic cataract groups. Blood glucose, lens turbidity, and apoptosis were measured. Lens epithelial cells were classified into the normal, blank, negative control (NC), *miR-211* mimics, *miR-211* inhibitors, siRNA-SIRT1, and *miR-211* inhibitors + siRNA-SIRT1 groups. *MiR-211*, Bcl-2, Bax, p53, and SIRT1 expressions of each group were detected. Cell proliferation, cycle and apoptosis were tested by MTT assay and flow cytometry. *MiR-211* can specifically bind to SIRT1 according to the luciferase system. SIRT1 protein concentration was strongly positive in normal mice and weakly positive in diabetic cataract mice. Apoptosis index of diabetic cataract mice was higher than the normal mice. Compared with normal mice, the expressions of *miR-211*, Bax, and p53 increased in diabetic cataract mice, while the Bcl-2 and SIRT1 expressions decreased. In comparison with the blank and NC groups, the expressions of *miR-211*, Bax, and p53 increased, while Bcl-2 and SIRT1 expressions decreased, and the proliferation decreased and apoptosis rate increased in the *miR-211* mimics and siRNA-SIRT1 groups; the results were contradicting for the *miR-211* inhibitor group. *MiR-211* could promote apoptosis and inhibit proliferation of lens epithelial cells in diabetic cataract mice by targetting SIRT1.

## Introduction

Cataract, an eye lens opacification, can lead to serious reversible visual impairment and blindness, and is a multifactorial disease caused by various factors, amongst which diabetes is an essential one [1,2]. Diabetes mellitus (DM) is an extensive chronic illness that affects over 285 million people worldwide and the figures are predicted to rise to 439 million by 2030 [3,4]. DM patients suffer from chronic complications with increasing morbidity and mortality; cataract and lens opacity are the earliest complications experienced by DM patients, which are characterized by severe metabolic disorders and high blood glucose level [5,6]. Clinical epidemiology and basic research have confirmed an association between diabetic retinopathy and cataract formation [4,7]. Lens epithelial cell apoptosis is a common cellular foundation for the development of non-congenital cataract in human beings and animals [8]. Former evidence revealed that high glucose concentrations could lead to apoptosis of human lens epithelial cell and inhibit proliferation [9]. MiRNA has been widely studied for its close association with lens epithelial cells [10–12].

MiRNA is a type of short non-coding RNA (approximately 18–23 nts), which acts as an evolutionarily conserved regulator of gene expression by pairing base-pairing with the 3′-UTR of the target mRNA [13]. Enough evidence has confirmed that miRNAs are often down-regulated in various cancers such as hepatocellular carcinoma and colon adenocarcinoma [14,15], and significantly affects diverse biological processes including proliferation, apoptosis, migration, invasion, and tumorigenesis [14]. MiRNAs have been identified in multiple ocular tissues, and they have a role in the development of lens and retina, ocular physiology, as well as many ocular diseases [16–19]. MiRNAs have been found to be differentially expressed in transparent and cataractous lens [20]. *MiR-211* belongs to a group of specific miRNAs that are highly expressed in human vitreous [21]. Silent information regulator (SIR2) family of genes, a highly conserved group of genes is present in the organism’s genomes and the encoded SIR proteins are involved in diverse processes from regulating gene silencing to DNA repairing [22]. Sirtulin 1 (SIRT1) has an affect on cell apoptosis, differentiation, and senescence, and the regulation of glucose and lipid metabolism [23]. SIRT1 as an NAD^+^-dependent deacetylase principally modulates downstream pathways of calorie restriction, which consequently has beneficial effects on glucose homeostasis [24]. Besides, SIRT1 has been observed to have a down-regulated expression in trigeminal sensory neurones in diabetic mice, and SIRT1 affects against cataract to some extent [25,26]. Until now, the mechanism of miRNA in diabetic cataract was not very well defined due the poorly obtained target gene information. Therefore, we hypothesized that SIRT1 could be a novel target gene of the miRNA member *miR-211* in diabetic cataract and the present study aimed at investgating the effects of *miR-211* on the proliferation and apoptosis of lens epithelial cells in diabetic cataract mice by regulating the *SIRT1* gene.

## Materials and methods

### Ethics statement

The animal experimental processes were approved by the Ethnic Committee of Shenzhen Eye Hospital, Ophthalmology College of Shenzhen University and conducted in strict accordance with the standards of the Guide for the Care and Use of Laboratory Animals published by the Ministry of Science and Technology of the People’s Republic of China in 2006.

### Experimental animals and model establishment

The present study included a total of 60 healthy male mice (25 ± 5 g), which were purchased from the Animal Experiment Center of Guangxi Medical University, Nanning, China. The mice were fed in separate cages at a temperature of 25°C and were exposed to light every 12 h; they were allowed to eat and drink without any restrictions. After 2 weeks of adaptive feeding and fasting for 12 h (but water), the experiment was conducted. No abnormalities of lens were observed under the slit-lamp microcamera (SL-3G, Topcon, Japan) before the experiment. The mice were divided randomly into the normal group (*n*=30) and model group (diabetic cataract group, *n*=30). Before establishing models, blood samples were collected from mice (fasted) of the normal and model groups via tail vein and the blood glucose level was determined using a blood glucose meter (U80, URIT Medical Co., Ltd., Guilin, China). Citric acid solution with 2% streptozotocin (STZ) (S0130, Sigma–Aldrich Chemical Co., St. Louis, MO, U.S.A.) was filtered through a 0.22-μm micropore. Mice in the model group were administered an intraperitoneal injection of STZ (50 mg/kg per time) [27]. Mice in the normal group were injected with the same amount of normal saline.

After standard feeding for 12 weeks, blood samples were collected from mice (fasted) in the normal and model groups via tail vein and the blood sugar was measured. The mice were dripped with 0.1 g/l tropicamide ophthalmic solution (jgtbka1, Jinan Jiage Biotechnology Company, Jinan, China) into the eyes, anesthetized with ether, and any changes in their lens were observed under a slit-lamp. It was graded according to the turbidity of the lens: grade I, the lens were clear and transparent without turbidity; grade II, the lens were slightly turbid with a small amount of vacuoles around; grade III, the lens were moderately turbid with vacuoles extending into the central area and haze turbidity appearing in the nuclei lentis; grade IV, the lens are highly turbid with vacuoles extending to the nuclear region as well as aggravated haze turbidity in the nuclei lentis; grade V, turbidity in the nuclei lentis developed into total cataract [28]. A diabetic cataract model was successfully established if the value of fasting blood glucose in the model group was over 14.0 mmol/l and the lens was turbid. The diabetic mice that survived and normal mice were anesthetized by an intraperitoneal injection containing 1–2 ml of 1% pentobarbital sodium (Shanghai Haling Biotechnology Co. Ltd., Shanghai, China) and were later killed by dislocating the cervical vertebra. The bilateral eyeballs of mice were extracted under a biological microscope (XSP-36; Shenzhen Boshida Optical Instrument Co., Ltd., Shenzhen, China). The eyeballs of the mice were then soaked in 250 U/ml saline three times under aseptic conditions (each time for 10 min) and placed in an ice bath; after which the cornea and iris were removed; crystalline lens were extracted and washed with physiological saline. The lens capsule was removed, placed in a 1.5-ml Ep cryovial, and stored in –80°C liquid nitrogen tank. All experimental procedures and animal use programs were performed with approval from the Animal Ethics Committee.

### Immunohistochemistry

The lens samples frozen at –80°C were extracted, fixed with 10% formalin solution, cut into serial sections (4 μm; some slices were used for TUNEL staining) and then embedded in paraffin. Tissue slices were placed in an incubator at 60°C for 1 h, after conventional xylene dewaxing and gradient alcohol dehydration, then the tissues were incubated with 3% H_2_O_2_ (BD5024; Bioworld Technology, Minneapolis, MN, U.S.A.) at a temperature of 37°C for 30 min, followed by a wash with PBS for four times for 2-min intervals. After 2 min of high-pressure antigen retrieval, these specimens were placed in 0.01 M citrate buffer with pH 6.0 and boiled at 95°C for 20 min, after which the slices were soaked in 3% H_2_O_2_ for 15 min to block the activity of peroxidase. Normal goat serum fluid (lot number: Ns01-01, Tyco Biotechnology Co., Ltd., Luoyang, China) was used to seal samples at a temperature of 37°C for 10 min. After the rabbit antimouse polyclonal antibody SIRT1 (bs-0921R, 1:500, Beijing Bioss Biotech Co. Ltd., Beijing, China) was added, the samples were placed at a temperature of 4°C for one night and washed with PBS. Then, the secondary antibody (bs-0921R-HRP, Beijing Bioss Biotech Co. Ltd., Beijing, China) labeled by horseradish peroxidase was added to the samples followed by incubation at room temperature for 30 min, coloring with DAB (CAS: 7411-49-6, Suzhou Industrial Park Yacoo Chemical Reagent Co., Ltd.) for 3 min and a rinse with water for 3 min. The samples were redyed with hematoxylin (Shanghai Bogoo Biotechnology Co., Ltd. Shanghai, China) for 20 s, rinsed under running water to clean any excess dye liquor and then sealed. The primary antibody was replaced by PBS as negative control and the pathological sections of glaucoma were set as positive control. These samples were observed and photographed under an optical microscope (XSP-36, Shenzhen Boshida Optical Instrument Co., Ltd., Shenzhen, China Shenzhen, China). Five views at high magnification (400×) were randomly selected in each slice. In each field, 100 cells were counted; positive cells >10% was considered as positive(+) and positive cells ≤10% as negative (–) [29]. The number of positive cells in each group was calculated in terms of mean ± S.D. in a percentage form.

### TUNEL staining

The prepared lens tissue slices were added into 3% H_2_O_2_ solution, allowed to rest at room temperature for 10 min, and washed with distilled water three times, each interval was 2 min. The slices were digested with protease K (20 μg/ml) (MB5088; Meilun Biotechnology, Dalian, China) at 37°C for 30 min and washed with PBS three times, 2 min each time. These sections were added into 3% H_2_O_2_ solution for 5 min to block the activity of endogenous peroxidase at room temperature, and washed with PBS three times, each interval was 2 min. After 0.1% citric acid with 0.1% Triton X-100 was added (FK-ml2089, Fanke Biotechnology Company, Shanghai, China), the samples were placed on ice for 4 min, washed with PBS three times, each time for 2 min. After adding 50-μl TUNEL mixed solution (ZK-8005, Beijing Zhongshan Golden Bridge Biotechnology Co., Ltd., Beijing, China), the samples were allowed to react at 37°C for 1 h, and washed with PBS three times, each time for 2 min. The samples were added with DAB/H_2_O_2_ color liquid (2014, Invitrogen Inc., Shanghai, China) at room temperature for 5 min, and the reaction was terminated by a wash with water, followed by hematoxylin redying, dehydration, transparency, and sealing. TUNEL staining showed that the apoptotic positive cells were dark brown in color with atrophied nucleus and chromatin gathering on the edge and endochylema was not stained. A total of five non-overlapping field visions were randomly and observed and accounted for under an optical microscope (XSP-36; Shenzhen Boshida Optical Instrument Co., Ltd., Shenzhen, China) to determine the TUNEL positive cell numbers in 100 lens tissues and the average value was selected after calculation. The positive apoptosis rate was presented by the percentage of apoptotic cells per unit area accounting for total cells [30].

### Quantitative real-time PCR

The total RNA of 100-mg lens tissues frozen at –80°C were extracted by MiRNeasy Mini Kit (217004, Qiagen Company, Hilden, Germany), and the concentration and purity of RNA were determined. TaqMan MicroRNA Assays Reverse Transcription Primer (4427975, Applied Biosystems Inc., U.S.A.) was used to convert RNA into cDNA by reverse transcription according to the instructions. The *miR-211*, SIRT1, Bcl-2, Bax, and p53 primers were designed and synthesized by TaKaRa Corporation (Takara Biotechnology Ltd., Dalian, China). (Table 1). ABI7500 quantitative PCR detector (7500, Applied Biosystems Inc., U.S.A.) was used for quantitative real-time PCR (qRT-PCR). The reaction conditions were: predenaturation at 95°C for 10 min, denaturation at 95°C for 10 s, annealing at 60°C for 20 s, extending at 72°C for 34 s, for a total of 40 cycles. The reaction system (20 μl): 10 μl SYBR Premix Ex TaqTM II, 0.8 μl PCR forward primer (10 μm), 0.8 μl PCR reverse primer (10 μm), 0.4 μl ROX reference dye, 2.0 μl cDNA template, and 6.0 μl sterile purified water. U6 was set as the internal reference for the relative expression of *miR-211* and β-actin for the relative expressions of SIRT1, Bcl-2, Bax, and p53; and 2^−ΔΔ*C*^_t_ indicated a ratio of gene expression between the experimental group and the control group, and the formula was as follows: ΔΔ*C*_T_ = Δ*C*_t_ (case group) – Δ*C*_t_ (control group), Δ*C*_t_ = *C*_t__miRNA_ – *C*_t__β-actin_. *C*_t_ was set as the number of amplification cycles before the real-time fluorescence intensity reached the set threshold. Each experiment was repeated thrice (mRNA expression was determined after 48 h of transfection with the same methods).

**Table 1:** Primer sequences for qRT-PCR

Genes	Primer sequences
*miR-211*	F: 5′-TCGGCAGGTCCCTTTGTCATCC-3′
	R: 5′-TGCAGGTCAACTGGTGTCGT-3′
*U6*	F: 5′-GCTTCGGCAGCACATATACTAAAAT-3′
	R: 5′- CGCTTCACGAATTTGCGTGTCAT -3′
*SIRT1*	F: 5′-GAACCTTTGCCTCATCTACATTTTG-3′
	R: 5′-CAAGTAAATAGTCTCAACGGTGGTT-3′
*Bcl-2*	F: 5′-CCGGGAGAACAGGGTATGA-3′
	R: 5′-CCTACCCAGCCTCCGTTAT-3′
*Bax*	F: 5′-AGATGAACTGGACAGCAATATG-3′
	R: 5′-CCTACCCAGCCTCCGTTAT-3′
*p53*	F: 5′-AAGACAGGCAGACTTTTCGCCACAG-3′
	R: 5′-GAAACTCCAAGCACAAACACGGA-3′
*β-actin*	F: 5′-ACCGTGGAGAAGAGCTACGA -3′
	R: 5′-GTACTTGCGCTCAGAAGGAG -3′

Abbreviations: F, forward; R, reverse.

### Western blotting

A total of 80 mg/kg frozen lens tissues (–80°C) were placed in a glass grinder and 1 ml of tissue lysate (BB-3209, BestBio, Shanghai, China) was added. The samples were placed in an ice bath and ground in order to obtain a homogenate, lysated with protein lysate at 4°C for 30 min, shaken once every 10 min and centrifuged for 20 min at 12000 revs/min at 4°C. The lipid layer was removed and the supernatant was extracted. BCA kit was used to determine the protein concentration of each sample (20201ES76, YeaSen Biotechnology Co. Ltd., Shanghai, China). Deionized water was added to adjust the loading quantity of a protein sample with 30-μg protein/lane. After preparing 10% SDS separation and concentration gels, tissues were mixed with sample buffer, boiled at 100°C for 5 min, followed by addition into each lane for electrophoretic separation using a microsampler after an ice bath and centrifugation; then the gel protein was transferred on to a nitrocellulose membrane. A total of 5% skim milk powder was used to seal nitrocellulose membrane at 4°C for one night. The diluted primary antibody was added: rabbit antimouse polyclonal antibody SIRT1 (bs-1921R, Beijing Bioss Biotech Co. Ltd., Beijing, China) (1:500), rabbit antimouse monoclonal antibody Bax (ab32503, Abcam Inc., Cambridge, MA, U.S.A.), rabbit antimouse polyclonal antibody Bcl-2 (bs-20351R, Beijing Bioss Biotech Co. Ltd., Beijing, China) (1:500), rabbit antimouse polyclonal antibody p53 (bs-8687R, Beijing Bioss Biotech Co. Ltd., Beijing, China) (1:500) and glyceraldehyde-3-phosphate dehydrogenase (GAPDH) (ab9485, Abcam Inc., Cambridge, MA, U.S.A.) (1:500) for overnight incubation and a wash with PBS three times at room temperature, each time for 5 min. Rabbit antimouse polyclonal antibody IgG labeled by horseradish peroxidase (HRP) was added and the tissues were shaken and incubated for 1 h at 37°C, washed with PBS three times, with 5 min intervals. Electrochemiluminescence (ECL) (ECL808-25, Biomiga Inc., U.S.A.) was mixed with nitrocellulose membrane at room temperature for 1 min. The liquid was extracted out, and then the tissues were covered with a plastic film for X-ray photography (36209ES01, Shanghai Qcbio Science & Technologies Co., Ltd. Shanghai, China) and observation. GAPDH was set as an internal reference; the proportion of gray value between the target band and reference band was set as the relative protein expression. Each experiment was repeated three times. Forty-eight hours after transfection, cells were collected with 100-μl cell lysate (BB-3203; BestBio, Shanghai, China), cooled in an ice bath at 4°C for 30 min, centrifuged for 20 min at 12000 revs/min and the supernatant was collected. The subsequent steps were the same as above.

### Cell culture

The anterior capsule of the frozen (–80°C) lens tissue was removed and sliced into pieces by a cutting needle. The tissues were added into Dulbecco’s modified Eagle’s medium (DMEM) low-glucose medium with 20% FBS (31600-034, Yanhui Biological Technology Co. Ltd, Shanghai, China), so as to make the capsular tissue slices scatter at the bottom of the bottle. Tissues were incubated at 37°C with 5% CO_2_ for 12–24 h. The DMEM culture medium with 100 ml/l bovine serum was added into the samples when the capsule membrane and the scattered lens epithelial cells grew adhering to the bottle, and the solution was changed every 3 days. The cells were subcultured until the bottom of the bottle was completely covered. Samples were washed once by D-Hanks solution (BTN100927, BOAO LAI Technology Co., Ltd., Beijing, China). The cells were added with 2.5 g/l trypsin (2 ml) and shaken for 2 min. After separating most of the cells from the bottom of the bottle, they were observed for contraction and separation from the bottle’s bottom under the inverted microscope, DMEM complete medium with 100 ml/l calf serum (BW120013, Biowit Technologies Co., Ltd., Shenzhen, China) was added; the cells were blown with a straw and subcultured (1:2).

### Cell grouping and transfection

The lens epithelial cells at logarithmic growth phase were adjusted to 10^7^/l in density, and inoculated into a six-well plate and 2-ml cell suspension solution was added to each hole. The cells were transfected when the cell density reached 30–50% according to the instructions of Lipofectamine 2000 introduction (1668019, Thermo Fisher Scientific, CA, U.S.A.). A total of 100 pmol *miR-211* mimics, *miR-211* 100 inhibitors, siRNA-SIRT1, *miR-211* inhibitors + siRNA-SIRT1, and negative control (the final concentration added into cells was 50 nm) were diluted by 250 μl serum-free Opti-MEM medium (31985, Gibco Company, U.S.A.), mixed gently and incubated at room temperature for 5 min. Lipofectamine 2000 (5 μl) was diluted with 250 μl serum-free Opti-MEM medium followed by incubation at room temperature for 5 min. The two samples were mixed, added into the culture hole, incubated at room temperature for 20 min, and cultured at 37°C for 6–8 h with 5% CO_2_, and replaced by a completely new medium (INV-00002, Wuxi Innovate Biomedical Technology Co., Wuxi, China). The subsequent experiments were conducted 24–48 h later. The cells were assigned into the normal group, blank group (without any transfection sequence), negative control (NC) group (transfected with *miR-211* negative control sequence), *miR-211* mimics group (transfected with *miR-211* mimics), *miR-211* inhibitors group (transfected with *miR-211* inhibitors), siRNA-SIRT1 group (transfected with siRNA-SIRT1), *miR-211* inhibitors + siRNA-SIRT1 group (transfected with *miR-211* inhibitors and siRNA-SIRT1).

### Dual luciferase reporter gene assay

The biological prediction website www.microRNA.org was employed to analyze the target genes of *miR-211*, and a dual luciferase reporter gene assay was performed to verify whether SIRT1 was a direct gene of *miR-211*. The full length of *SIRT1* gene at 3′-UTR region (F: GCGCTCGAGTTGTTCCACCAGCATTAG; R: GCGCGGCCGCCATTAATTTAACATTC) were cloned and extended into the pmirGLO (E1330, Promega Corporation, Madison, WI, U.S.A.) Luciferase vector named pSIRT1-Wt. Site-directed mutagenesis method was conducted using a bioinformatics software to predict the binding site of *miR-211* and its target gene *SIRT1*. The pSIRT1-mut vector was established, with pRL-TK vector (E2241, Promega Corporation, Madison, WI, U.S.A.) of luciferase as the internal reference. *MiR-211* mimics and *miR-211* NC were respectively transfected with luciferase reporter vector into HEK-293T cells (CRL-1415, American Type Culture Collection (ATCC), U.S.A.). A fluorescence detector was used for detecting the florescence intensity (lot number: Glomax20/20, Promega Corporation, Madison, WI, U.S.A.) [31].

### MTT assay

After 48 h of transfection, the cells were collected, cultured with RPMI 1640 medium containing 10% FBS (61870-127, Gibco Company, U.S.A.) to form a cell suspension of 2.5 × 10^5^/ml, which was inoculated in a 96-well plate (eight holes in each group, 100 μl in each hole according to the experimental grouping). The samples were placed in a incubator at 37°C with 5% CO_2_ and the culture plate was withdrawn after 24, 48, and 72 h. A total of 10 μl of 5 mg/ml MTT solution was added followed by cell culture for 4 h. After the supernatant was extracted, 100 μl DMSO (D5879-100ML, Sigma–Aldrich Chemical Co., St. Louis, MO, U.S.A.) was added into tissues and mixed for 10 min so as to dissolve the formazan crystals produced by live cells. The optical density (OD) value of each hole at 490 nm site was measured using a microplate reader (BS-1101, Germany Iron Experiment Equipment Co. Ltd., Nanjing, China). Each experiment was repeated thrice. The cell viability curve was protracted with the time point set as the abscissa and the OD value as the ordinate.

### Flow cytometry

#### PI single staining

After 48 h of transfection, the cells were collected, washed with cold PBS for three times, and centrifuged. The supernatant was discarded; the cells were resuspended in PBS, adjusted to a density of approximately 1 × 10^5^ cells/ml, and fixed with 1 ml 75% ethanol (–20°C precooled) at 4°C for 1 h. After centrifuging the cells, the ice ethanol was discarded and the cells were rinsed with PBS to abandon the supernatant. Approximately 100 μl of RNase A (GE101-01, Beijing TransGen Biotech Co., Ltd., Beijing, China) was added and the cells were kept in a water bath at 37°C for 30 min devoid of light, stained with 400 μl protease inhibitor (PI) (88378, Sigma–Aldrich Chemical Co., St. Louis, MO, U.S.A.) and mixed for an even mixture. At 4°C for 30 min devoid of light, the cell cycle was determined by detecting red fluorescence at the excitation wavelength of 488 nm with flow cytometry (CytoFLEX, Beckman Coulter, CA, U.S.A.).

#### Annexin V/PI double staining

After 48 h of transfection, the cells were digested by 0.25% EDTA-free trypsin (YB15050057, Yu Bo Biological Technology Co., Ltd., Shanghai, China) and collected in the flow tube. The supernatant was discarded after centrifugation. The cells were washed with cold PBS thrice and centrifuged after which the supernatant was discarded. Annexin-V-FITC/PI dye liquor was prepared in the ratio 1:2:50 in a mix containing Annexin-V-FITC, PI, and HEPES solution according to the instructions of Annexin-V-FITC kit (K201-100, BioVision, U.S.A.). Approximately 1 × 10^6^ cells were resuspended with 100 μl dye liquor, incubated for 15 min, and added in 1 ml HEPES (PB180325, Procell, Wuhan, China). The FITC and PI were determined, respectively with 525 and 620 nm band pass filter at the wavelength of 488 nm, and the cell apoptosis was detected. The experiment was repeated thrice.

### Statistical analysis

SPSS 21.0 statistical software (SPSS, Inc., Chicago, U.S.A.) was used for data analysis and all data were represented by mean value ± S.D. One-way factor ANOVA was applied for comparing amongst multiple groups and *t* test was employed for two groups. *P*<0.05 was considered to be significantly different.

## Results

### Blood glucose concentration measurement

Eight weeks after the experiment, only 27 mice survived in the model group with a 90% survival rate whereas all the mice in the normal group survived. The highest value of fasting blood glucose in normal mice was 14.0 mmol/l, but in the model group it peaked to (20.34 ± 3.31) mmol/l, which was significantly higher than that observed in the normal group (*P*<0.05) (Table 2). This was a clear indication of successful diabetic models establishment. According to the turbidity of the lens, the mice in the normal group were classified as Grade I: the lens were clear and transparent without turbidity; in the model group, the lens of the mice showed turbidity with different degrees including Grade I, Grade II, Grade IV, and Grade V. The mice with turbidity of Grade III accounted for (54.45 ± 3.21)%, significantly higher than that in Grades I, II, IV, and V (Table 3), suggesting that cataract mice model was successfully established.

**Table 2:** Blood glucose concentration in normal mice and diabetic cataract mice

Blood glucose concentration	Normal mice (*n*=30)	Diabetic cataract mice (*n*=27)	*P*
Before modeling (mmol/l)	3.74 ± 0.41	3.81 ± 0.75	0.659
After modeling (mmol/l)	4.34 ± 1.05	20.34 ± 3.31	<0.001

**Table 3:** Turbidity detection of lens between the normal mice and diabetic cataract mice

Turbidity grade	Normal mice	Diabetic cataract mice	*P*
I (%)	100 ± 0	4.45 ± 1.21	<0.001
II (%)	0 ± 0	21.15 ± 1.21	<0.001
III (%)	0 ± 0	54.45 ± 3.21	<0.001
IV (%)	0 ± 0	12.25 ± 1.08	<0.001
V (%)	0 ± 0	7.82 ± 1.78	<0.001

### SIRT1 protein expression decreased in lens tissue of mice in the model group

Immunohistochemistry results showed that the negative cells were blue and purple; the weak positive cells were light yellow, whereas the strongly positive cells were chocolate brown. SIRT1 positive substance was located in the nuclear cytoplasm of a lens cell and the expression of SIRT1 protein was observed in the lens tissue of mice in the model group and normal group. SIRT1 protein showed a strong positive expression in mice lens tissue in the normal group (52.12 ± 5.52)% compared with the weak positive expression in the model group (18.31 ± 1.88)%. In comparison with the normal mice, SIRT1 protein level significantly decreased in lens tissue in the model group (*P*<0.05) (Figure 1).

**Figure 1:** Expression of SIRT1 protein of lens tissue in mice in the normal and model groups (200×) (**A**) Comparison of SIRT1 protein expression of lens tissue in the normal and model groups by immunohistochemistry; (**B**) comparison of the positive expression rates of SIRT1 protein in the normal and model groups; *, *P*<0.05 compared with the normal group.

### Apoptosis index of lens tissues increased in the model group

TUNEL staining showed that cells with brown nucleus were apoptotic and those with blue nucleus were negative. Apoptosis index value of lens tissue in normal mice was (3.01 ± 0.25)%, while in the diabetic cataract mice was (18.37 ± 1.56)%. Compared with the normal group, apoptosis index in the model group significantly increased (*P*<0.05) (Figure 2).

**Figure 2:** Cell apoptosis of lens tissue in the normal and model groups (400×) (**A**) Cell apoptosis of lens tissue in the normal and model groups; (**B**) comparison of apoptosis index in the normal and model groups; *, *P*<0.05 compared with the normal group. Abbreviation: AI, apoptosis index.

### Expressions of *miR-211*, SIRT1, Bcl-2, Bax, and p53 in lens tissues of mice in the normal and model groups

In the diabetic cataract group, *miR-211* expression and mRNA expressions of Bax and p53 significantly increased (*P*<0.05) and the mRNA expressions of SIRT1 and Bcl-2 obviously decreased (*P*<0.05) compared with the normal group (Figure 3A). Western blotting showed that protein expressions of Bax and p53 increased (*P*<0.05), protein expressions of SIRT1 and Bcl-2 significantly decreased (*P*<0.05) in the diabetic cataract group in comparison with the normal group (Figure 3B,C).

**Figure 3:** Expression of *miR-211* and mRNA and protein expressions of SIRT1, Bcl-2, Bax, and p53 in lens tissues of mice (**A**) *miR-211* expression and mRNA and protein expressions of SIRT1, Bcl-2, Bax, and p53 in mice lens; (**B**) strip chart of SIRT1, Bcl-2, Bax, and p53 proteins; (**C**) expressions of SIRT1, Bcl-2, Bax, and p53 proteins in mice lens; *, *P*<0.05 compared with the normal group.

### *miR-211* specifically targeted SIRT1

According to the results from biological website www.microRNA.org, SIRT1 was the target gene of *miR-211* (Figure 4A). To verify if SIRT1 is the direct target gene of *miR-211*, luciferase reporter vector wild-type-*miR-211*/SIRT1 and mutant-*miR-211*/SIRT1 recombinant plasmids were added with 3′-UTR wild sequence of SIRT1 after which a mutation sequence was established. Luciferase system showed that compared with the NC group, the luciferase signal of wt-*miR-211*/SIRT1 transfection group decreased significantly (*P*<0.05), while no significant difference was observed in the luciferase signal of mut-*miR-211*/SIRT1 plasmid group (*P*>0.05) (Figure 4B). Therefore, it can be concluded that *miR-211* can specifically bind to the *SIRT1* gene.

**Figure 4:** The verification of the targetting relationship between *miR-211* and SIRT1 (**A**) Sequence of 3′-UTR region of *SIRT1* mRNA binding with *miR-211*; (**B**) luciferase activity detection; *, *P*<0.05 compared with the NC group.

### *miR-211* expression and mRNA expressions of SIRT1, Bcl-2, Bax, and p53 in each group

In comparison with the normal group, the expressions of *miR-211*, Bax, and p53 in the other groups increased prominently, while the expressions of SIRT1 and Bcl-2 decreased significantly (*P*<0.05). Compared with the blank and NC groups, the *miR-211* expression in the *miR-211* mimics group increased (*P*<0.05); there was no significant change in the *miR-211* expression in the siRNA-SIRT1 group (*P*>0.05); the mRNA expressions of Bax and p53 in the *miR-211* mimics and siRNA-SIRT1 groups increased (*P*<0.05); the mRNA expressions of SIRT1 and Bcl-2 decreased significantly (*P*<0.05). In the *miR-211* inhibitors group, the *miR-211* expression and the mRNA expressions of Bax and p53 decreased, while the SIRT1 and Bcl-2 expression significantly increased; the *miR-211* expression in the *miR-211* inhibitors + siRNA-SIRT1 group decreased but there were no obvious changes in the expressions of Bax, p53, SIRT1, and Bcl-2 (*P*>0.05). There was no significant difference between the blank group and NC group (*P*>0.05) (Figure 5).

**Figure 5:** Relative mRNA expressions of *miR-211*, Bax, p53, SIRT1, and Bcl-2 in each group *, *P*<0.05 compared with the normal group; ^#^, *P*<0.05 compared with the blank and NC groups.

### Expressions of SIRT1, Bcl-2, Bax, and p53 proteins in each group

In comparison with the normal group, an increase in the protein expressions of Bax and p53 and a decrease in the expressions of SIRT1 and Bcl-2 was observed in the blank group, NC group, *miR-211* mimics group, *miR-211* inhibitors group, siRNA-SIRT1 group, and *miR-211* inhibitors + siRNA-SIRT1 group (*P*<0.05). Compared with the blank and NC groups, the expressions of Bax and p53 proteins in the *miR-211* mimics and siRNA-SIRT1 groups increased (*P*<0.05), while the expressions of SIRT1 and Bcl-2 decreased (*P*<0.05); the protein expressions of Bax and p53 in the *miR-211* inhibitors group decreased and the expressions of SIRT1 and Bcl-2 increased (*P*<0.05); no significant change was observed in the protein expressions of SIRT1, Bcl-2, Bax, and p53 in the *miR-211* inhibitors + siRNA-SIRT1 group (*P*>0.05). No significant difference was observed between the blank group and NC group (*P*>0.05) (Figure 6).

**Figure 6:** The protein expressions of SIRT1, Bcl-2, Bax, and p53 in each group (**A**) The protein strip chart; (**B**) the relative protein expression in seven groups; *, *P*<0.05 compared with the normal group; ^#^, *P*<0.05 compared with the blank and NC groups.

### Changes of cell proliferation after transfection

No significant difference in cell viability was detected in each group during the 24th h after transfection (*P*>0.05), while the difference was observed during the 48th h. In comparison with the normal group, the cell proliferation activity decreased significantly in the other groups (*P*<0.05). In comparison with the blank group and NC group, cell proliferation activity in the *miR-211* mimics group and siRNA-SIRT1 group decreased while cell proliferation in the *miR-211* inhibitors group increased appreciably (*P*<0.05). No significant changes in cell proliferation were observed in the *miR-211* inhibitors + siRNA-SIRT1 group (*P*>0.05). In comparison with the *miR-211* inhibitors group, the proliferation activity in the *miR-211* inhibitors + siRNA-SIRT1 group decreased remarkably (*P*<0.05) (Figure 7).

**Figure 7:** Proliferation of lens epithelial cells in seven groups *, *P*<0.05 compared with the normal group; ^#^, *P*<0.05 compared with the blank and NC groups; ^&^, *P*<0.05 compared with the *miR-211* inhibitors group.

### Cell-cycle distribution and apoptosis after transfection

PI single staining showed the cell percentages in the blank group, NC group, *miR-211* mimics group, *miR-211* inhibitors group, siRNA-SIRT1 group, and *miR-211* inhibitors + siRNA-SIRT1 group significantly increased in the G_0_-phase, but decreased in S-phase and G_2_-phase (*P*<0.05) in contrast with the normal group. Compared with the blank group and NC group, the cell percentage in the G_1_-phase increased significantly in the *miR-211* mimics group and siRNA-SIRT1 group while being decreased at S-phase and G_2_-phase (*P*<0.05); the cell percentage in the *miR-211* inhibitors group significantly declined at G_1_-phase, but increased at S- and G_2_-phases (*P*<0.05); no obvious changes in cell percentages were observed in G_1_-, S-, and G_2_-phases in the *miR-211* inhibitors + siRNA-SIRT1 group (*P*>0.05). The cells percentage in G_1_-phase was increased significantly but decreased in S- and G_2_-phases in the *miR-211* inhibitors + siRNA-SIRT1 group was higher compared with the value observed in the *miR-211* inhibitors group (*P*<0.05) (Figure 8).

**Figure 8:** Detection of cell cycles by flow cytometry (**A**) Distribution curves of cell cycles in each group; (**B**) cell cycles in seven groups; *, *P*<0.05 compared with the normal group; ^#^, *P*<0.05 compared with the blank and NC groups; ^&^, *P*<0.05 compared with the *miR-211* inhibitors group.

Double Annexin V/PI double staining showed that in comparison with the normal group the apoptosis rate in the blank group, NC group, *miR-211* mimics group, *miR-211* inhibitors group, siRNA-SIRT1 group, and *miR-211* inhibitors + siRNA-SIRT1 group increased significantly (*P*<0.05). The apoptosis rate in the *miR-211* mimics group and siRNA-SIRT1 group increased (*P*<0.05) though it declined in the *miR-211* inhibitors group (*P*<0.05). Compared with the blank group and NC group, no apparent changes were observed in the apoptosis rate in the *miR-211* inhibitors + siRNA-SIRT1 group (*P*>0.05). The apoptosis rate in the *miR-211* inhibitors + siRNA-SIRT1 group was higher than the *miR-211* inhibitors group (*P*<0.05) (Figure 9). Lower right quadrant exhibited early metaphase apoptotic cells while the upper right quadrant was a representation of the late apoptotic cells and secondary necrotic cells. The upper left quadrant presented cells with mechanical injury or necrotic cells, and the lower left quadrant represented living cells.

**Figure 9:** Detection of cell apoptosis by flow cytometry in seven groups (**A**) Cell apoptosis chart; (**B**) apoptotic cell number in seven groups; *, *P*<0.05 compared with the normal group; ^#^, *P*<0.05 compared with the blank and NC groups; ^&^, *P*<0.05 compared with the *miR-211* inhibitors group.

## Discussion

STZ has been used as a diabetes-inducing agent in various animal species in the past three decades due to its induction of clinical properties in different animal species similar to those associated with diabetes in humans [32]. In our study, we investigated the influence of *miR-211* on the proliferation and apoptosis of lens epithelial cells in diabetic cataract mice by targetting the *SIRT1* gene. Our results mainly demonstrated that inhibiting the *miR-211* expression could diminish the rate of apoptosis of lens epithelial cells in diabetic cataract mice whereas silencing the *SIRT1* gene could stimulate the rate of apoptosis of lens epithelial cells in diabetic cataract mice. Meanwhile, our study also proved that the inhibition of *miR-211* expression could upsurge the expression of anti-apoptotic protein Bcl-2 of lens epithelial cells in diabetic cataract mice.

The qRT-PCR results indicated that *miR-211* was highly expressive in lens epithelial cells of diabetic cataract mice and SIRT1 was weakly positive and was not highly expressed in the model group compared with the normal group. Various miRNAs depicted unique tissue- and stage-specific expression patterns, which was a clear indication of their potential functions in retina and other ocular tissues [33]. Mutations in miRNAs or their target RNAs could potentially lead to a series of retinal abnormalities [34]. It has been indicated from the qRT-PCR results that *miR-29a* expression obviously increased in 2- and 4-week diabetic rat tissues [8]. Various miRNAs have been observed to exhibit ocular enrichment, including *miR-211* [35]. An overexpression of SIRT1 was observed in atherosclerotic plaques in type 2 diabetic subjects [36]. It has been reported that SIRT1 activation can intensify mitochondrial function and prolong the survival of mice with a high-calorie diet [37–39]. SIRT1 transgenics display has been acknowledged to improve glucose tolerance as a result of decrease in the production of hepatic glucose and increase in adiponectin levels. Functional gain of SIRT1 in prime organisms can aid in metabolic adaptation to insulin resistance and decrease the overall body energy requirements [40,41]. In the present study, we observed a higher *miR-211* expression and lower SIRT1 expression in diabetic mice than normal mice. A previous study reported that miRNAs play a role in the regulation of expression of their downstream target genes [42]. Our study proved that *miR-211* could specifically bind to the *SIRT1* gene regions by dual luciferase reporter gene assay. The exact mechanism underlying how *miR-211* affects lens epithelial cells in diabetic cataract mice by targetting *SIRT1* gene needs to be studied in depth in the future.

Additionally, our results found that *miR-211* could inhibit the proliferation of lens epithelial cells and promote cataract development by suppressing the expression of *SIRT1* gene. A previous study also confirmed that *miR-22* could inhibit cell proliferation by targetting the 3′-UTR of SIRT1 in glioblastoma could inhibit cell proliferation and *miR-22*-SIRT1 pathway was a potential target for glioblastoma treatment [43]. Our study showed that *miR-211* could promote the apoptosis of lens epithelial cells via targetting *SIRT1* gene. It has been reported that high glucose concentration can lead to apoptosis of human lens epithelial cells [9]. Some recent research studies demonstrated that apoptosis of lens epithelial cells was in a close relationship with cataract formation, and death of lens epithelial cells was caused due to cataractogenic stress disarranged homeostasis which consequently leads to oxidation and hydration that contributed to cataract formation [44,45]. A previous study suggested that cancer cells could be killed by miR-induced apoptosis and the killed cells were disposed of by lymphocytic destruction and proteolysis [46]. Likewise, the study showed that in comparison with the normal group, the apoptosis index of the lens tissues increased significantly in the diabetic cataract group, which clearly indicated that *miR-211* could promote the apoptosis of lens epithelial cells in diabetic cataract mice.

In our study, we observed that inhibiting the *miR-211* expression could stimulate the expression of anti-apoptotic protein Bcl-2 in lens epithelial cells of diabetic cataract mice. A recent study demonstrated that expression of *miR-211* increased after down-regulating the level of Bcl-2 [47]. The Bcl-2 expression up-regulated in tissues after transfection of *miR-21* mimics and expression of Bax, apoptosis, caspase-3 activity, and the chemosensitivity decreased, indicating *miR-21* could promote Bcl-2 expression by combining with the 3′-UTR of Bcl-2 [48]. Likewise, our study showed that *miR-211*-induced Bcl-2 up-regulation was linked to apoptosis of diabetic cataract cells. One study detected that the *miR-211* expression in colorectal cancer tissues decreased the apoptosis of colorectal cancer cells by stable gene transfection technology [49]. In addition, we observed that in comparison with the blank and NC groups, expressions of Bax and p53 proteins increased in the *miR-211* mimics and siRNA-SIRT1 groups, while they decreased in the *miR-211* inhibitors group. The p53 protein is protected against rapid degradation largely as a result of post-translational modifications and activated p53 protein allowed it to up-regulate gene expressions that promote exit from the cell cycle or that which favor apoptosis [22]. Milne et al. [24] demonstrated that SIRT1 activators could decrease the acetylation state of p53, a well-known SIRT1 substrate. SIRT1 can regulate glucose/lipid metabolism via its deacetylase activity on multiple substrates [41]. Vaziri et al. [22] also reported that acetylated p53 peptide could serve as a substrate for SIR2α and p53 de-acetylation by mammalian SIR2 which is specific and does not result from indiscriminate deacetylase functions.

To conclude, our observations demonstrated that *miR-211* was highly expressed in lens epithelial cells of diabetic cataract mice, and it participated in the regulation of cell apoptosis and proliferation by targetting *SIRT1* gene. Thus, *miR-211* might be a novel underlying target for the treatment of diabetic cataract. However, since retinal acid content was not measured due to the limited funds and time, further experiments on retinal tissues are required for detailed studies in the future.

## Abbreviations

DM: diabetes mellitus
DMEM: Dulbecco’s modified Eagle’s medium
GAPDH: glyceraldehyde-3-phosphate dehydrogenase
NC: negative control
OD: optical density
PI: protease inhibitor
qRT-PCR: quantitative real-time PCR
SIR2: silent information regulator
SIRT1: sirtulin 1
STZ: streptozotocin
